# Relationship between Resting Pulse Rate and Lipid Metabolic Dysfunctions in Chinese Adults Living in Rural Areas

**DOI:** 10.1371/journal.pone.0049347

**Published:** 2012-11-07

**Authors:** Chong-jian Wang, Yu-qian Li, Lin-lin Li, Ling Wang, Jing-zhi Zhao, Ai-guo You, Yi-rui Guo, Wen-jie Li

**Affiliations:** 1 Department of Epidemiology and Biostatistics, College of Public Health, Zhengzhou University, Zhengzhou, Henan, PR China; 2 Research Centre, CHU Sainte-Justine, Montreal, Quebec, Canada; 3 Department of Clinical Pharmacology, School of Pharmaceutical Science, Zhengzhou University, Zhengzhou, Henan, PR China; 4 Department of Endocrinology, Military Hospital of Henan Province, Zhengzhou, Henan, PR China; 5 Department of Disease Control and Prevention, Henan Provincial Center for Disease Control and Prevention, Zhengzhou, Henan, PR China; Nihon University School of Medicine, Japan

## Abstract

**Background:**

Resting pulse rate has been observed to be associated with cardiovascular diseases. However, its association with lipid metabolic dysfunctions remains unclear, especially resting pulse rate as an indicator for identifying the risk of lipid metabolic dysfunctions. The purpose of this study was to examine the association between resting pulse rate and lipid metabolic dysfunctions, and then evaluate the feasibility of resting pulse rate as an indicator for screening the risk of lipid metabolic dysfunctions.

**Methods:**

A cross-sectional survey was performed, and 16,926 subjects were included in this study from rural community residents aged 35–78 years. Resting pulse rate and relevant covariates were collected from a standard questionnaire. The fasting blood samples were collected and measured for lipid profile. Predictive performance was analyzed by receiver operating characteristic (ROC) curve.

**Results:**

A significant correlation was observed between resting pulse rate and TC (*r* = 0.102, *P* = 0.001), TG (*r* = 0.182, *P* = 0.001), and dyslipidemia (*r* = 0.037, *P* = 0.008). In the multivariate models, the adjusted odds ratios for hypercholesterolemia (from 1.07 to 1.15), hypertriglyceridemia (1.11 to 1.16), low HDL hypercholesterolemia (1.03 to 1.06), high LDL hypercholesterolemia (0.92 to 1.14), and dyslipidemia (1.04 to 1.07) were positively increased across quartiles of resting pulse rate (*P* for trend <0.05). The ROC curve indicated that resting pulse rate had low sensitivity (78.95%, 74.18%, 51.54%, 44.39%, and 54.22%), specificity (55.88%, 59.46%, 57.27%, 65.02%, and 60.56%), and the area under ROC curve (0.70, 0.69, 0.54, 0.56, and 0.58) for identifying the risk of hypercholesterolemia, hypertriglyceridemia, low HDL hypercholesterolemia, high LDL hypercholesterolemia, and dyslipidemia, respectively.

**Conclusion:**

Fast resting pulse rate was associated with a moderate increased risk of lipid metabolic dysfunctions in rural adults. However, resting pulse rate as an indicator has limited potential for screening the risk of lipid metabolic dysfunctions.

## Introduction

Previous studies have shown that resting pulse rate is associated with the development of cardiovascular diseases, and elevated resting pulse rate is an important indicator of increased morbidity and mortality among people with hypertension, coronary artery disease, and diabetes mellitus [1]–[5]. A recent epidemiological study has shown that resting pulse rate is associated with an increased risk of metabolic syndrome [6]. However, relatively few studies have evaluated the correlation between resting pulse rate and the risk of lipid metabolic dysfunctions, particularly in rural adults. In addition, no study has explored whether resting pulse rate could be used as an indicator to identify the risk of lipid metabolic dysfunctions in rural adults.

Lipid metabolic dysfunction is a widely recognized risk factor for cardiovascular diseases, which is the leading cause of death in both developed and developing countries [7], [8]. The World Health Organization (WHO) estimates that lipid metabolic dysfunctions are associated with more than half of global cases of ischemic heart disease and more than four million deaths per year [9]. Emerging evidence demonstrates that lipid metabolic dysfunctions can be prevented and controlled, which will be helpful to reduce morbidity and mortality of cardiovascular diseases and other relevant diseases [10], [11]. Therefore, identifying relevant factors that may predict the risk of lipid metabolic dysfunction is an important approach toward improved understanding and prevention of this disease, especially within high-risk population [12]. We examined the correlation between resting pulse rate and the risk of lipid metabolic dysfunctions in a large-scale epidemiological survey of rural Chinese adults. We also evaluated the feasibility of resting pulse rate as an indicator for screening the risk of lipid metabolic dysfunctions.

**Table 1:** Characteristics of study population stratified by resting pulse rate (n = 16,926).

Variables	Resting pulse rate, beats/min				*P* value
	≤67 (n = 4,341)	68–74 (n = 4,517)	75–81 (n = 3,946)	>81 (n = 4,122)	
Age (years), mean (±sd)	52.87 (10.80)	52.78 (10.83)	53.28 (10.86)	54.70 (11.23)	0.001
Female, n (%)	2,033 (46.83)	2,771 (61.35)	2,619 (66.37)	2,895 (70.23)	0.001
Education, n (%)					0.001
No education	680 (15.66)	823 (18.22)	688 (17.44)	815 (19.77)	
Primary school	1,471 (33.89)	1,556 (34.45)	1,342 (34.01)	1,483 (35.98)	
Middle school	1,748 (40.27)	1,696 (39.36)	1,553 (36.36)	1,498 (36.34)	
High school or more	442 (10.18)	442 (9.79)	363 (9.20)	326 (7.91)	
Marital status, n (%)					0.020
Married/cohabitation	3,940 (90.83)	4,113 (91.12)	3,621 (91.79)	3,699 (89.78)	
Divorced/widowed/unmarried	401 (9.17)	404 (8.88)	325 (8.21)	423 (10.22)	
Physical activity, n (%)					0.001
Low	1,185 (27.30)	1,376 (30.46)	1,253 (31.75)	1,447 (35.10)	
Moderate	874 (20.13)	1,002 (22.18)	858 (21.74)	894 (21.69)	
High	2,282 (52.57)	21.39 (47.35)	1,835 (46.50)	1,781 (43.21)	
Mean individual income (annual), n (%)					0.057
<1000 CNY	1,763 (40.61)	1,730 (38.30)	1,496 (37.91)	1,637 (39.71)	
1000 ∼ CNY	1,347 (31.03)	1,429 (31.64)	1,252 (31.73)	1,331 (32.29)	
≥2000 CNY	1,231 (28.36)	1,353 (30.06)	1,198 (30.36)	1,154 (28.00)	
Current smoking, n (%)	1,204 (27.74)	955 (21.14)	733 (18.58)	674 (16.35)	0.001
Current drinking, n (%)	584 (13.45)	482 (10.67)	368 (9.33)	345 (8.37)	0.001
More high-fat diet, n (%)	214 (4.93)	252 (5.58)	225 (5.70)	238 (5.77)	0.298
More vegetable and fruit intake, n (%)	2,235 (51.81)	2,264 (50.12)	1,964 (49.77)	2,030 (49.30)	0.101
Family history of hypercholesterolemia, n (%)	422 (9.72)	468 (10.36)	416 (10.54)	461 (11.18)	0.104
Waist circumference (cm), mean (±sd)	82.45 (9.70)	83.26 (10.06)	83.57 (10.42)	84.98 (10.82)	0.001
Pulse pressure (mmHg), mean (±sd)	46.30 (13.84)	46.88 (12.95)	48.28 (12.77)	51.30 (13.30)	0.001
Glucose (mmol/L), mean (±sd)	5.46 (1.08)	5.57 (1.22)	5.78 (1.65)	6.06 (2.02)	0.001
TC (mmol/L), mean (±sd)	4.46 (0.90)	4.58 (0.93)	4.57 (0.92)	4.62 (0.99)	0.001
TG (mmol/L), mean (±sd)	1.61 (1.09)	1.68 (1.13)	1.76 (1.19)	1.82 (1.25)	0.001
HDL-C (mmol/L), mean (±sd)	1.18 (0.26)	1.17 (0.26)	1.16 (0.26)	1.15 (0.27)	0.001
LDL-C (mmol/L), mean (±sd)	2.57 (0.75)	2.64 (0.77)	2.60 (0.76)	2.60 (0.81)	0.001
Hypercholesterolemia, n (%)	157 (3.62)	216 (4.78)	185 (4.69)	265 (6.43)	0.001
Hypertriglyceridemia, n (%)	707 (16.29)	817 (18.09)	823 (20.86)	941 (22.83)	0.001
Low HDL hypercholesterolemia, n (%)	1,356 (31.43)	1,472 (32.59)	1,316 (33.35)	1,416 (34.35)	0.033
High LDL hypercholesterolemia, n (%)	68 (1.57)	80 (1.77)	55 (1.39)	90 (2.18)	0.040
Dyslipidemia, n (%)	1,798 (41.42)	1,972 (43.66)	1,805 (45.74)	1,905 (46.22)	0.001

**Abbreviations:** sd, standard deviation; CNY: China Yuan; TC  =  total cholesterol; TG  =  triglyceride s; HDL  =  high density lipoprotein; LDL  =  low density lipoprotein.

## Methods

### Subjects

A population-based cross-sectional survey was performed, and subjects were selected randomly from eligible candidates listed in the residential registration record from rural district in Henan Province. The eligibility of the candidate was defined as those who were stable residents for at least 10 years in the areas aged 35–78 years, and were free from the following conditions: 1) severe psychological disorders, physical disabilities, cancer, chronic kidney disease, Alzheimer’s disease, or dementia, within 6 months; or 2) currently diagnosed with tuberculosis, acquired immune deficiency syndrome (AIDS), and other infectious diseases. After cancer (n = 48), chronic kidney disease (n = 152), physical disabilities (n = 8), tuberculosis (n = 12), and other infectious diseases (n = 9) were excluded, 17,042 subjects who met the criteria were enrolled in the study. Of the eligible participants, 116 (0.68%) subjects were excluded because of missing information on resting pulse rate (n = 69), lipid profile (n = 47). Ultimately, 16,926 subjects were selected for the present analysis. The procedure of the study was approved by the Zhengzhou University Medical Ethics Committee, and written informed consent was obtained from all participants.

**Table 2:** Odds ratios and 95% confidence intervals of lipid metabolic dysfunctions according to quartiles of resting pulse rate (n = 16,926).

Variables	Resting pulse rate, beats/min				*P* for trend
	≤67 (n = 4,341)	68–74 (n = 4,517)	75–81 (n = 3,946)	>81 (n = 4,122)	
**Hypercholesterolemia**					
Crude *OR*(95%*CI*)	1.00	1.06(0.93–1.20)	1.10(1.03–1.18)	1.14(1.05–1.22)	0.001
Adjusted *OR*(95%*CI*) *	1.00	1.07(0.93–1.22)	1.12(1.04–1.20)	1.15(1.07–1.23)	0.001
**Hypertriglyceridemia**					
Crude *OR*(95%*CI*)	1.00	1.09(1.02–1.17)	1.14(1.10–1.18)	1.15(1.11–1.20)	0.001
Adjusted *OR*(95%*CI*) *	1.00	1.11(1.04–1.18)	1.14(1.09–1.17)	1.16(1.12–1.20)	0.001
**Low HDL hypercholesterolemia**					
Crude *OR*(95%*CI*)	1.00	1.02(0.99–1.05)	1.03(1.01–1.05)	1.05(1.02–1.08)	0.006
Adjusted *OR*(95%*CI*) *	1.00	1.03(1.01–1.07)	1.05(1.02–1.07)	1.06(1.03–1.10)	0.005
**High LDL hypercholesterolemia**					
Crude *OR*(95%*CI*)	1.00	0.92(0.77–1.11)	1.10(1.01–1.18)	1.11(1.01–1.19)	0.018
Adjusted *OR*(95%*CI*) *	1.00	0.92(0.78–1.08)	1.12(1.04–1.20)	1.14(1.08–1.18)	0.012
**Dyslipidemia**					
Crude *OR*(95%*CI*)	1.00	1.03(1.00–1.06)	1.04(1.02–1.06)	1.05(1.03–1.08)	0.009
Adjusted *OR*(95%*CI*) *	1.00	1.04(1.01–1.07)	1.05(1.03–1.07)	1.07(1.04–1.10)	0.006

* Adjusted for age, sex, education, marital status, individual income, smoking, drinking, fat intake, vegetable and fruit intake, family history of hypercholesterolemia, central obesity, physical activity, pulse pressure and medication use.

### Measurement of Pulse Rate and Covariates

Pulse rate and blood pressure were measured by electronic sphygmomanometer (Omron HEM-770A, Japan) in the sitting position three times. During the process of measurement, a standardized protocol was adapted from procedure recommended by the American Heart Association [13]. Participants were advised to avoid alcohol, cigarette smoking, coffee, tea, and excessive exercise for at least 30 minutes prior to having their pulse rate and blood pressure read.

Relevant covariates that might be expected to affect pulse rate and lipid metabolic dysfunctions were selected and collected using a standard questionnaire administered by trained staff, including of demographic characteristics (age and sex), socioeconomic status (educational level, marital status, and individual annual income), family and individual disease history (hypertension, diabetes, heart disease, cancer, chronic kidney disease, stroke, tuberculosis, and AIDS), and dietary and lifestyle (smoking, drinking, fat intake, vegetable and fruit intake, and physical activity). Body weight and height were measured twice in light indoor clothing without shoes to the nearest 0.1 kg and 0.1 cm, respectively. Waist circumference (WC) was measured twice at the mid-point between the lowest rib and the iliac crest to the nearest 0.1 cm, after inhalation and exhalation. Central obesity based on WC (Male: WC≥90 cm; Female: WC≥80 cm) was defined according to WHO criteria for the Asia-Pacific population [14]. The interview included questions related to the diagnosis and treatment of hypercholesterolemia. All data were collected by specially trained physicians and public health workers using standardized methods with stringent levels of quality control.

An overnight fasting blood specimen was collected in a vacuum tube containing EDTA for measurement of lipid profile. Blood specimens were centrifuged at 4°C and 3000 rpm for 10 minutes, and the plasma was transferred and stored at −20°C for biochemical analyses. Total cholesterol (TC), triglycerides (TG), and high-density lipoprotein cholesterol (HDL-C) were analyzed enzymatically by automatic biochemical analyzer (Hitachi 7080, Tokyo, Japan) with use of commercial reagents. Low-density lipoprotein cholesterol (LDL-C) level was calculated by use of the Friedewald equation for participants with TG level <4.52 mmol/L (400 mg/dl): LDL-C = TC-(HDL-C)-TG/5 [15].

### Ascertainment of Outcomes

Lipid metabolic dysfunctions were defined as a self-reported history of hypercholesterolemia and undiagnosed dyslipidemia. Lipid metabolic dysfunctions in participants without a prior diagnosis of hypercholesterolemia were categorized according to the China Adult Dyslipidemia Prevention Guide (2007 Edition) criteria as follows [16]: hypercholesterolemia was defined as the level of TC ≥6.22 mmol/L (240 mg/dl); hypertriglyceridemia was defined as the level of TG ≥2.26 mmol/L (200 mg/dl); low HDL hypercholesterolemia was defined as the level of HDL-C <1.04 mmol/L (40 mg/dl); and high LDL hypercholesterolemia was defined as the level of LDL-C ≥4.14 mmol/L (160 mg/dl). The subjects were considered as dyslipidemia if one of TC, TG or HDL-C were dysfunctions based on the above diagnostic criteria. All study participants were asked to bring their prescription medications during the clinic visit. A self-reported history of hypercholesterolemia was confirmed by the use of hypolipidemic agents (AHFS code: 24: 06.04, 24: 06.05, 24: 06.06, 24: 06.08, 24: 06.92). In addition, the hospital charts of all hospitalized cases of hypercholesterolemia were reviewed.

### Statistical Analysis

For statistical analysis, in order to facilitate comparison with previously reports, values of resting pulse rate were stratified into quartile: Quartile 1 (Q_1_≤67 beats/min), Quartile 2 (Q_2_ 68–74 beats/min), Quartile 3 (Q_3_ 75–81 beats/min), and Quartile 4 (Q_4_>81 beats/min). For continuous variables, differences groups were determined by one-way ANOVA. Categorical variables were evaluated using Mantel-Haenszel statistics of chi-square (χ*^2^*) test, and the trend chi-square test was used to measure the dose-response relationship. The Pearson correlation coefficient was used to analyze the linear association between resting pulse rate and lipid metabolic dysfunctions. Univariate and multivariate logistic regression models were built to quantify the risk of lipid metabolic dysfunctions adjusting for possible confounders and socioeconomic variables. Covariates included age (continuous), sex (two categories), education level (four categories), marital status (two categories), individual income (three categories), smoking (yes *vs.* no), drinking (yes *vs.* no), fat intake (two categories), vegetable and fruit intake (two categories), family history of hypercholesterolemia (yes *vs.* no), physical activity (three categories), waist circumference (two categories), pulse pressure (two categories), and medications use (yes *vs.* no). Receiver Operating Characteristic (ROC) curve was used to assess predictive performance using the same data with multivariate logistic regression analysis. Area under ROC curve (AUC) was also utilized to compare the combined sensitivity and specificity among different categories of the subjects. All analyses were conducted using SAS 9.1 (SAS Institute, USA). All reported *P*-values were two-sided, and *P*-values less than 0.05 were considered to be statistically significant.

**Table 3:** Predictive performance of resting pulse rate to screen lipid metabolic dysfunctions in rural adult subjects (n = 16,926).

	Sensitivity (%, 95% CI)	Specificity (%, 95% CI)	PPV (%, 95% CI)	NPV (%, 95% CI)
Hypercholesterolemia	78.95 (66.12–88.59)	55.88(53.17–58.45)	6.77 (5.73–8.84)	98.54 (96.85–99.01)
Hypertriglyceridemia	74.18 (67.78–79.89)	59.46 (56.67–62.21)	24.01 (21.41–27.38)	93.02 (89.01–96.13)
Low HDL hypercholesterolemia	51.54 (46.81–56.22)	57.27 (54.12–60.44)	35.56 (31.28–40.98)	72.04 (67.52–77.82)
High LDL hypercholesterolemia	44.39 (39.18–47.33)	65.02 (62.45–68.89)	47.45 (43.18–50.79)	62.86 (59.25–65.78)
Dyslipidemia	54.22 (50.11–58.26)	60.56 (57.22–63.93)	48.89 (48.10–56.12)	65.61 (59.14–65.93)

## Results

Table 1 shows the baseline characteristics of study population stratified by resting pulse rate. In general, age, waist circumference, pulse pressure, and glucose level were higher, and lipid metabolic dysfunctions risk factors such as lower-educational level, divorced or widowed, positive family history of hypercholesterolemia, less physical activity and vegetable and fruit intake, and more high-fat diet were more prevalent among subjects with higher resting pulse rate. Current smoking and drinking were inversely related to pulse rate (Z = −13.10 and −7.87, *P*<0.01). The prevalence of hypercholesterolemia, hypertriglyceridemia, low HDL hypercholesterolemia, high LDL hypercholesterolemia, and dyslipidemia is significantly increased with higher resting pulse rate (Z = 1.64–45.36, *P*<0.01).

A statistical relationship was observed between resting pulse rate and TC (*r* = 0.102, *P* = 0.001), TG (*r* = 0.182, *P* = 0.001), and dyslipidemia (*r* = 0.037, *P* = 0.008), but the correlation coefficient is weak. Although a negative correlation was detected between resting pulse rate and HDL-C (*r* = −0.026, *P* = 0.322), it was not statistically significant. In addition, no significant relationship existed between resting pulse rate and LDL-C (*r* = 0.026, *P* = 0.321).

Table 2 summarizes the unadjusted and adjusted odds ratios and 95% confidence interval of lipid metabolic dysfunctions according to quartiles of resting pulse rate. The results showed that resting pulse rate was positively associated with the risk of lipid metabolic dysfunctions through a dose-response effect (*P* for trend <0.05). When adjusted for age, education, marital status, individual income, smoking, drinking, fat intake, vegetable and fruit intake, family history of hypercholesterolemia, central obesity, physical activity, pulse pressure, and medication use, the adjusted odds ratios for hypercholesterolemia (from 1.07 to 1.15), hypertriglyceridemia (1.11 to 1.16), low HDL hypercholesterolemia (1.03 to 1.06), high LDL hypercholesterolemia (0.92 to 1.14), and dyslipidemia (1.04 to 1.07) were significantly increased across quartiles of resting pulse rate for rural adults.

Table 3 presents the optimum sensitivity, specificity, positive predictive value (PPV), and negative predictive value (NPV) for resting pulse rate to screen lipid metabolic dysfunctions in rural adults. The results indicated that resting pulse rate as an indicator has relatively low sensitivity and specificity for identifying the risk of hypercholesterolemia (78.95% sensitivity and 55.88% specificity), hypertriglyceridemia (74.18% and 59.46%), low HDL hypercholesterolemia (51.54% and 57.27%), high LDL hypercholesterolemia (44.39% and 65.02%), and dyslipidemia (54.22% and 60.56%) at the optimum cut-off point values, respectively. Further analysis showed that resting pulse rate has limited potential for screening an increased risk of hypercholesterolemia (AUC = 0.70±0.04, 95% *CI*: 0.68–0.72), hypertriglyceridemia (AUC = 0.69±0.02, 95% *CI*: 0.66–0.71), low HDL hypercholesterolemia (AUC = 0.54±0.02, 95% *CI*: 0.51–0.56), high LDL hypercholesterolemia (AUC = 0.56±0.02, 95% *CI*: 0.55–0.57), as well as dyslipidemia (AUC = 0.58±0.02, 95% *CI*: 0.56–0.61).

## Discussion

There were two fundamental questions that were answered in this study: 1) whether a relationship exists between resting pulse rate and lipid metabolic dysfunctions, and 2) whether resting pulse rate could be used as an indicator for screening the risk of lipid metabolic dysfunctions in rural adults.

Firstly, the study analyzed the correlation coefficient between resting pulse rate and lipid metabolic dysfunctions. The results showed that a statistical relationship was detected between resting pulse rate and TC (*r* = 0.102), TG (*r* = 0.182), and dyslipidemia (*r* = 0.037), but no significant correlation was observed with HDL-C (*r* = −0.026) and LDL-C (*r* = 0.026). Previous results from American and Israeli Industries Study supported our findings [17]–[19]. In addition, similar relationships were also observed between resting pulse rate and lipid metabolic dysfunctions by Freitas and his colleagues [20], but the correlation was weaker than results from their study (TC: *r* = 0.189, TG: *r* = 0.215, HDL-C: *r* = 0.035, and LDL-C: *r* = 0.118). Alternatively, univariate regression analyses showed that resting pulse rate was positively associated with risk of lipid metabolic dysfunctions through dose-response effect (*P* for trend <0.05). After adjusting for possible confounders, similar results were also observed by multivariate logistic regression analysis. This finding was generally in agreement with a previous study, and fast resting pulse rate was positively associated with an increased risk of hypertriglyceridemia [21]. However, the positive association between resting pulse rate and lipid metabolic dysfunctions was not found in a Japanese study [22], but a dose-response effect was observed between resting pulse rate and lipid metabolic dysfunctions in their study, which was similar to our findings. The reason for this could be explained by the different ethical, racial, or geographic background.

Previous studies showed that resting pulse rate provides an overall index of autonomic tone, and elevated resting pulse rate may reflect an imbalance in the autonomic nervous system favouring sympathetic activation [23], [24]. Enhanced sympathetic activity has been linked to lipid metabolic dysfunctions, high blood pressure, insulin sensitivity, and the metabolic syndrome [18], [25]–[27]. Our findings support the biological plausibility of a positive association between resting pulse rate and lipid metabolic dysfunctions.

Secondly, this study considered accuracy performance by examining discrimination. Sensitivity and specificity are important when testing whether a predictor can accurately discriminate positive and negative outcomes [28]. The ideal indicator should have both high sensitivity and high specificity [29], [30]. The results showed that resting pulse rate as an indicator has low sensitivity and specificity for identifying true positive or negative patients in rural adults. Since AUC provides a superior performance index in addition to superior accuracy, it is often used to evaluate the predictive accuracy of classifiers [31], [32]. This study also used AUC values for performance comparisons of different levels of resting pulse rate. The results indicated that resting pulse rate has limited potential for screening an increased risk of lipid metabolic dysfunctions. The results were similar to those of a recent published study from Brazilian population [20]. Overall, our findings suggested that resting pulse rate as an indicator for identifying the risk of lipid metabolic dysfunctions had fairly poor accuracy and reliability.

Although this study was the first to evaluate the correlation between resting pulse rate and lipid metabolic dysfunctions in rural adults, some limitations should be noted. The cross-sectional design does not offer support to causality statements and, therefore, prospective studies from different populations are necessary to describe more accurately the longitudinal relationship between resting pulse rate and lipid metabolic dysfunctions. Secondly, the results were based on a sample design and, hence, incorporating multi-center data should be considered in future research. Thirdly, only resting pulse rate was used to identify those at high risk of lipid metabolic dysfunctions in this study, and combination with other cardiovascular risk factor could screen more adequately subjects at increased risk to develop lipid metabolic abnormalities [5]. In addition, the absence of insulin measures to screen more clearly the relationship between resting pulse rate and glucose metabolism should be considered in future research [20]. Another possible limitation is that the cut-off of resting pulse rate was defined using quartile [33]. This approach was chosen because resting pulse rate stratified into quartiles has been applied in most previously epidemiological studies [3], [5], [20]; this allowed us to compare our results with previously published reported. Despite these limitations, the results are based on a large population-based epidemiologic study after adjusting for potential confounders, and the exposure assessment of resting pulse rate has been carried out systematically in this study, which precludes differential reporting in relation to the outcome.

### Conclusion

In summary, our findings demonstrated that fast resting pulse rate was associated with a moderate increased risk of lipid metabolic dysfunctions in rural adults, and that fast pulse rate at rest might raise the risk for the development of lipid metabolic dysfunctions. In addition and more importantly, this data revealed that resting pulse rate as an indicator has limited potential for screening an increased risk of lipid metabolic dysfunctions, which suggested that resting pulse rate might not be utilized as a perfect risk indicator of lipid metabolic dysfunctions in rural adults.
